# Environmental Policy Selection and Town Resident Satisfaction Assessment: Under Governance of Localism

**DOI:** 10.1155/2022/4932712

**Published:** 2022-09-30

**Authors:** Kuo-Yan Wang, Jing Yu, Chia-Yang Ning

**Affiliations:** School of Economics and Management, Guangdong University of Petrochemical Technology, Maoming, China

## Abstract

Upper authorities have tightly controlled local budgets, especially at the administrative township level. Taiwan has been facing this particular phenomenon for a long period. This article explains how a township, before general elections, sees the choice of an improved environmental administrative work plan as a political advantage and uses simple and easy-to-use collective decision-making to assist. Then, survey residents' perceptions of implementing the new environmental policy. The research results are discussed not only as suggestions to improve the effectiveness of township public environmental policies and to respond to the needs of civilians appropriately but also to lead future research directions.

## 1. Introduction

The state determines all taxes, although many countries have developed new administrative measures that reconcile public services and funding while also considering the fairness of fiscal transfers, such as the introduction of specific local charges. For example, Horvat et al. [1] found that Slovenia's local governments could not raise public services funds. Nonetheless, Kirchgässner [2] argues that a stronger central government with a high degree of integration of administrative resources appears to increase the probability of ending the integration event in the context of high financial reliance on central government financing. However, this possibility can also easily lead to stagnation of local investment, especially in the absence of external funding [1]. As a result, public service resources lack professional governance and flexibility. In 2005, the Slovenian government amended the Financing of Municipalities Act. The five years following these amendments are worthy of attention—specifically, their impact on intergovernmental relationships and citizens' satisfaction with the loose budget allocation policy. For example, increasing the debt at the municipal level has even derived from the common phenomenon of “budget federalism” [3, 4].

A similarly interesting phenomenon has also occurred in Taiwan. The regional-level government revenue and expenditure expanded dramatically from 2010 to 2014, in which numerous county-level governments upgraded to a special municipal level because of public administrative and organizational reforms. The supreme administrative authority of Taiwan has granted extended powers to the local governments within 14 municipalities and 6 special municipalities. According to polls regarding citizen satisfaction with Taiwanese mayors, the chief administrative officers of the municipalities that had access to more financial resources did not always achieve the highest rankings. The lowest-ranked mayors predominantly came from regions affected or controlled by local political factions [5]. As the strategic selection of appropriate policies is the key to winning over voters, local administrative authorities must prioritize practical and essential issues for their residents instead of spending lavishly on projects just for face value.

In the previous discussion on this issue, very little literature discusses this issue in depth. Therefore, this empirical study attempts to reveal township governments' environmental administrative work factors that stimulate voter support before the general election. This study involved field-level governments adopting a multicriteria decision-making approach (MCDM) in selecting focused environmental administrative work options. Then, half a year after the policy was implemented, a survey was conducted among the residents of the interviewed townships to survey perceptions of the new policy. The findings yielded several interesting results, particularly regarding the personal dynamics of township leaders in pushing for new administrative work policies. In addition, the phenomenon of “buying policy votes” has also been scrutinized.

This case study is aimed at solving the best township-level environmental administrative policy implementation system. Public administration problem-solving generally requires grasping principles that are easy to understand and use [6–8]. To this end, the ideal solution similarity ranking technique (TOPSIS) is introduced in this work rather than the commonly used qualitative decision-making techniques e.g., the Delphi, forced group discussion. We then analyze the results of resident satisfaction surveys in the case of the township and other highly homogeneous townships that have not implemented the new policy.

The following part introduces the TOPSIS to the problem of local administrative policy solution selection. Secondly, through descriptive statistical analysis, compare the differences in the satisfaction of township residents before and after the implementation of the new environmental policy, and discuss related phenomena. The final section concludes our findings.

## 2. TOPSIS-Selecting an Appropriate Policy in a Simple Way

Most optimization methods utilized in decision-making have been introduced as a response to the optimal solution to study a variety of administrative situations. However, simple and easy-to-use methods are still less discussed in environmental administration. TOPSIS was proposed by Chen and Hwang [9] and extended by Hwang and Yoon [10]. The rationale for the method is the option of the chosen choice closest to the ideal solution; the closer the two are the better. The main assumption of this model is to help decision makers avoid finding the maximum deviation from the negative ideal value (worst solution), and when the value is closer to the positive ideal value, it is the optimal solution [11]. The technique has been successfully applied to environmental improvement strategies [12], mass transportation fuel selection [13], large project solutions [14], highway bus route selection [15], and even at contributions for regional economic revitalization [16], as well as artwork surveys [17].

The TOPSIS procedure consists of the following six steps:

1. Integrate the normalized decision matrix. The normalized value *r*_*ij*_ is calculated as

(1) r=ijfij/Σj=1j,fij2,j=1,⋯,J,i=1,⋯n.

(2) Measure the weighted normalized decision matrix. The normalized weighted value *v_ij_* is calculated as

(2) $$\begin{array}{c} v_{ij}=w_{i}r_{ij},j=1,\cdots J;i=1,\cdots ,n, \end{array}$$

where *w_i_* is the weight of the *i*th attribute or criterion and *w*_*i*_ = 1

(3) Define the ideal and negative-ideal solution

(3) $$\begin{array}{c} A^{*}=\left\{{{\text{v}}_{i}}^{*},\cdots ,{v_{n}}^{*}\right\}=\left\{\left(\text{j}\max\left.v_{ij}\right|i\in I^{\prime }\right),\left(j\min\left.v_{ij}\right|i\in I^{\prime \prime }\right)\right\}, \end{array}$$

(4) $$\begin{array}{c} A^{-}=\left\{{{\text{v}}_{i}}^{-},\cdots ,{v_{n}}^{-}\right\}=\left\{\left(j\min\left.v_{ij}\right|i\in I^{\prime }\right),\left(j\max\left.v_{ij}\right|i\in I^{\prime \prime }\right)\right\}, \end{array}$$

where *I′* is associated with benefit criteria and *I^”^* is associated with cost criteria

(4) Determine the separation measures using the *n*-dimensional Euclidean distance. The separation of each alternative from the ideal solution is given as

(5) $$\begin{array}{c} D_{\text{j}}^{*}=\sqrt{\overset{n}{\underset{i=1}{\sum }}{\left(v_{ij}-v_{i}^{*}\right)}^{2}},j=1,\cdots ,J. \end{array}$$

Similarly, the separation from the negative-ideal solution is given as

(6) $$\begin{array}{c} D_{\text{j}}^{-}=\sqrt{\overset{n}{\underset{i=1}{\sum }}{\left(v_{ij}-v_{i}^{-}\right)}^{2}},j=1,\cdots ,J. \end{array}$$

(5) Calculate the relative closeness to the ideal solution. The proximity of the solution *a*_*j*_ concerning *A*^∗^ is defined as

(7) $$\begin{array}{c} C_{\text{j}}^{*}=\frac{D_{j}^{-}}{\left(D_{j}^{*}+D_{j}^{-}\right)},j=1,\cdots ,J. \end{array}$$

(6) Finally, rank the preference order

### 2.1. An Empirical Case

#### 2.1.1. TOPSIS in Policy Selection

Township B has about 130,000 residents. As a satellite town near City A, it has a convenient transportation network and superior living functions. With a general election approaching, the current mayor of township B is fighting for re-election. In addition to implementing the previous political ideas, Town B's management must propose quick-acting short-term policy plans as a selling point to attract voters. After repeated arguments, four new policy options were offered as follows: increasing the number of parks, the number of libraries, the number of free shuttle buses, or the number of waste disposal routes. Administrative professionals and scholars jointly participated in the final choice based on township B's financial situation and expected residents' satisfaction (Table 1). Each data was collected in government public information (Table 2) based on the currently available budget and expected future fiscal policy. In the initial assessment of the weights of the various criteria, the relevant decision-making experts were government officials in the finance sector, members of the B township council, and public administration scholars.

Experts attempted to unearth the results through interviewing the results of a pair of questionnaires from the Analytical Hierarchy Process (AHP), giving some weight to the relative importance of each criterion, and are presented in Table 3. The most significant criteria for evaluating proposed new policy options are those that directly benefit residents, according to citizens' attitudes toward the management performance of incumbent townships. In addition, the expected budget support is also the focus of implementing the new policy; that is to say, the government's fiscal revenue and expenditure are also the focus of the expert group's consideration.

Table 4 shows the weighted normalized decision matrix Eq. (2).

For determining the optimal solution, the next is utilized by Eq. (3) and (4), the results that *A*^∗^ = {0.068, 0.088, 0.089, 0.009, 0.014, 0.031};  *A*^–^ = {0.025, 0.011, 0.002, 0.052, 0.059, 0.083}. Then, this study employed Eq. (5) and (6) to measure the separation of each solution from the ideal solution (Table 5).

Finally, Table. 6 indicates that the added garbage disposal routes at township B are the optimal solution for implementing a new environmental policy.

#### 2.1.2. Descriptive Analysis Results

The researchers surveyed the township inhabitants joining the garbage disposal route policy in township B on January 1, 2022, observing the residents' satisfaction before and after the new policy. From July 1 to July 15, 2022, townships A, B, and C in the same municipal district were surveyed. Among them, townships A and C did not introduce new environmental policies. This study personally distributed 804 random questionnaires to the three surveyed township inhabitants who chose cluster sampling. After excluding unwilling and invalid respondents, 756 valid respondents (*n* = 756, about 94%) remained.

During the pretest phase from July 15 to July 31, each subdimension was from respondents' opinions. The administration performance design of township B managers has four components: public attention, regional development, policy satisfaction, and confidence in a future administration. We utilized a Likert 1 (extremely agree) to 5 (extremely disagree) rating scale. The questionnaire design considered reliability and validity (Cronbach′s alpha value = 0.7). Bartlett's test was lower than 0.01, meaning higher significance, and the KMO value was 0.24. Each item reflects a list of selected topics with a significant difference of 5%.  Table 7 shows that the respondents in township B were most recognized with the administrative satisfaction (79%) of the locality.

## 3. Discussions

Three parts will be discussed in this section. First, the benefits of the township-level government utilizing TOPSIS as an optimal group decision-making tool are described in the solution selection problem. Second, dynamic information is introduced along with the routing garbage collection truck of township B—the addition of the garbage disposal routes—which had the new policy implemented, unlike the previous static information. Finally, this study emphasizes an adverse phenomenon: policy vote buying at the local administrative level and existing coping strategies.

### 3.1. Simplifying the Policymaking

People's values, opinions, knowledge, abilities, and political systems influence policymaking. This diversity is destined to often conflict with each other, and different perspectives are often overlooked in decision-making. For the empirical cases of township election-driven decision-making procedures, resistance, or more complex situations often occur in the joint decision-making ways due to the interests of each faction. The TOPSIS method can help decision makers consider comprehensive alternatives and make better choices because it is introduced in this paper and can fully refer to the opinions of experts and representatives. In this way, even if there are differences between the decision-making options, they still focus on the problem.

### 3.2. A Powerful Promotional Tool for the Incumbent Township Mayor's Exposure

Unlike other areas where garbage is cleared and transported at designated locations, in Taiwan, due to the implementation of the policy of “no garbage on the ground”, the government's environmental department is responsible for most garbage removal work. Garbage collection trucks will appear in residential areas daily to collect and process garbage.

Further, Taiwan is the world's reputable producer of light-emitting diodes (LEDs). [18]. Many garbage trucks in Taiwan's township cleaning unit install LED display boards to replace previous banner strip installations. Traditionally, the banner strip contains government propaganda in static form on the garbage trucks utilized by the daily routine township garbage disposal service. The new pattern uses an LED display board to illustrate the dynamic public information.

Interestingly, the most noted is that the personal mark of the incumbent mayor is presented with the dynamic public information while the garbage disposal truck is going through its route rather than only being presented at the township office. The incumbent mayor is receiving full publicity with the new policy of adding garbage truck disposal routes. The survey revealed that the exposure of the incumbent mayor as a potential candidate for the next election had shown significant increases.

### 3.3. Avoiding ‘Policy Vote Buying' and Strengthening Administrative Efficiency

As the survey revealed, it is worth mentioning that the attitudes of residents from township B toward the incumbent mayor are higher than in other towns where the new policy was not implemented as effectively as in township B. Can this kind of administrative work, especially in the preelection period, be considered policy vote buying? In general, Schaffer [19] defined “vote buying” as “In offering money, goods, or services selectively there are, broadly speaking, three ways in which givers might hope to get recipients to vote, or not vote, for a particular candidate.”; Markovic [20] mentioned this phenomenon is easy to be manipulated by populism and social intervention, and it lacks long-term policy planning. Understandably, such behavior is against the law in countries or regions where free elections are implemented. Scholars have also pointed out that the township-level administrative works usually pay attention to visible items because of its policy scope approaching citizens directly [21]. In practical terms, township managements do everything possible to satisfy the demands and needs of the voter (i.e., if voters ask for a favor), even beyond the scope of the law. The only way for the voter to reciprocate is by voting for the candidate they deem the most responsive. Undoubtedly, beef politics impeded the normalization of the local administration.

To eliminate the drawbacks of vote-buying policy at the township level, the Taiwanese authorities restructured the local government during 2010-2014 in the four special municipalities: New Taipei, Taoyuan, Taichung, and Tainan. The changes to Taipei and Kaohsiung's two original special municipalities, commonly known as the “six metropolitans” (Liu du). Under the new municipalities, each township has become a district, and a district governor assigned by the upper authorities has replaced the existing township mayor. The original local representative assembly was integrated into the superior municipal council. Compared with the special municipality, only 36.4% of the overall annual budget in Taiwan can be assigned to the municipality and township government. The greatest advantage of these newly upgraded municipalities is tax redistribution, which accounted for 64.6% in 2015 [22]. A primary concern is whether the follow-up administrator at the district level can effectively shut down policy vote-buying.

Some other concerns regarding administrative efficiency arise when the original township administration transforms into a district administration under the new special municipality. This transformation changes the local political ecology and weakens the policy vote-buying phenomenon. A notable example occurred in Tainan, where a newly upgraded municipality suffered a deadly dengue fever outbreak between August and September 2015. Mosquitos predominantly spread this virus, is more likely to spread in hot weather, and may cause high fevers, headaches, itching, and joint pain [23]. At the onset of such an epidemic, a township authority can take immediate countermeasures such as fumigating, setting up a quarantine area, or providing vaccines. A district authority must first report the epidemic situation to the disease control center of the municipality. The center will then decide which measures to take. Opinion polls revealed that when the municipality administration officials of Tainan did not respond rapidly to the outbreak, satisfaction with the mayor declined (Taipei [24]). Changes to a municipality designation denote that a township acquires more financial resources. The rapid response of a municipality—in this case, spending available money on urgent needs—is a significant factor in resident satisfaction. As local administrative units are in close contact with residents, effective management of public funds is undoubtedly an issue of paramount importance for current local administrations.

## 4. Conclusions

Unlike other qualitative decision-making assistance methods, this study views the TOPSIS approach as a township-level preselection policy recommendation that plays an important role in MCDM by experts, scholars, and township representatives. Through exploratory case studies, despite cultural or geographical differences, this study explores new policies to increase waste disposal routes, which can help township management and residents' daily lives. The survey results showed that township residents agreed with the latest environmental policy. Further, many of the implications led describe dynamic public information, including the current mayor's markings, while being displayed on routing garbage trucks and increasing visibility.

This study focuses on addressing policy-based vote buying at the township level and workarounds to address this phenomenon, but its follow-up effects remain to be seen. Future research could investigate whether higher-level local governments effectively avoided policy votes before elections and discover more convenient simple techniques used in environmental decisions. These questions are worthy of further exploration.

## Figures and Tables

**Table 1:** Evaluation of hierarchical structure for new policy solution selection.

Goal	Solution	Criteria
The optimal solution of strengthening the township office administrative work	Add the numbers of community park	Expected expenditure budget
	Add the numbers of library	Expected increase in public income
	Add the routes of free shuttle bus	Expected upper government grants
	Add the garbage disposal routes	Expected tax redistribution
		Expected self-fundraising
		Expected directly benefit the residents

**Table 2:** Collected data from each criterion.

Criteria	Solution			
	Add the number of community parks	Add the number of libraries	Add the routes of the free shuttle bus	Add the garbage disposal routes
Expected expenditure budget (Mn)	18.37	22.76	8.43	18.45
Expected increase in public income (Mn)	0.74	0.51	1.13	4.12
Expected upper government grants (Mn)	3.22	5.12	0.21	8.38
Expected tax redistribution (Mn)	9.81	4.73	1.87	6.66
Expected self-fundraising (Mn)	1.05	3.16	4.49	2.35
Expected directly benefit the residents (per 1,000 person)	7.23	10.44	12.68	19.53

**Table 3:** Criteria weights.

Criterion	Financial sector	Elected representative assemblies	Academic scholar	Average
Expected expenditure budget	0.2762	0.1984	0.1334	0.2027
Expected increase public income	0.1839	0.1098	0.1240	0.1392
Expected upper government grants	0.1998	0.1898	0.1498	0.1798
Expected tax redistribution	0.1081	0.1393	0.1201	0.1225
Expected self-fundraising	0.1234	0.1022	0.2090	0.1449
Expected directly benefit the residents	0.1086	0.2605	0.2637	0.2109

**Table 4:** Normalized matrix.

Solution	Criteria					
	Expected expenditure budget	Expected increase public income	Expected upper government grants	Expected tax redistribution	Expected self-fundraising	Expected directly benefit the residents
Add park numbers	0.054	0.016	0.034	0.052	0.014	0.031
Add library numbers	0.068	0.011	0.054	0.025	0.041	0.031
Add free shuttle bus routes	0.025	0.024	0.002	0.009	0.059	0.054
Add garbage disposal routes	0.055	0.088	0.089	0.035	0.031	0.083

**Table 5:** Separation measure of each alternative.

Cj1^∗^	0.069	Cj1^–^	0.058
Cj2^∗^	0.064	Cj2^–^	0.059
Cj3^∗^	0.089	Cj3^–^	0.037
Cj4^∗^	0.043	Cj4^–^	0.088

**Table 6:** TOPSIS ranking results.

Solution	Rank	Index
Add park numbers	3	0.457
Add library numbers	2	0.479
Add free shuttle bus routes	4	0.294
Add garbage disposal routes	1	0.671

**Table 7:** The administrative performance survey result.

	Administrative satisfaction				Public attention				Local construction				Confidence in future development			
	Satisfied		Unsatisfied		Attention		Ignore		Good		No-good		Confidence		Unconfidence	
Township A incumbent mayor (*n*_1_ = 271)	(144)	53%	(73)	27%	(125)	46%	(43)	16%	(119)	44%	(57)	21%	(149)	55%	(70)	26%
Township B incumbent mayor (*n*_2_ = 263)	(208)	79%	(32)	12%	(190)	72%	(13)	5%	(179)	68%	(26)	10%	(189)	72%	(29)	11%
Township C incumbent mayor (*n*_3_ = 222)	(129)	58%	(31)	14%	(102)	46%	(16)	7%	(107)	48%	(25)	11%	(120)	54%	(53)	24%

## Data Availability

The data used to support the findings of this study are included within the article.
